This article has been retracted.

# Injectable hydrogel encapsulating Cu_2_MnS_2_ nanoplates for photothermal therapy against breast cancer

**DOI:** 10.1186/s12951-018-0409-3

**Published:** 2018-10-27

**Authors:** Ji-jun Fu, Ming-yue Chen, Jie-xia Li, Jun-hua Zhou, Sheng-nan Xie, Ping Yuan, Bo Tang, Cheng-cheng Liu

**Affiliations:** 1 Department of Medical Oncology, The Fifth Affiliated Hospital of Guangzhou Medical University, Guangzhou Medical University, Guangzhou, 510700 China; 2 Key Laboratory of Molecular Target & Clinical Pharmacology, School of Pharmaceutical Sciences, Guangzhou Medical University, Guangzhou, 511436 China; 3 Department of Biochemistry and Molecular Biology, Medical College of Shantou University, Shantou, 515041 Guangdong Province China; 4 School of Pharmaceutical Sciences, China Pharmaceutical University, No. 639 Longmian Avenue, Jiangning District, Nanjing, 211198 Jiangsu China; 5 School of Pharmacy, Nantong University, No. 19 Qixiu Road, Nantong, 226001 Jiangsu Province China

**Keywords:** Cu_2_MnS_2_, Nanoplates, Hydrogel, Thermosensitive, Injectable, In-situ, Photothermal

## Abstract

**Background:**

In order to explore the possibility of treating breast cancer by local photo-therapy, a photothermal agents loaded in situ hydrogel was established. In detail, The Cu_2_MnS_2_ nanoplates were prepared by one-pot synthesis and, the thermosensitive Pluronic F127 was used as the hydrogel matrix. The Cu_2_MnS_2_ nanoplates and the hydrogel were characterized by morphous, particle size, serum stability, photothermal performance upon repeated 808 nm laser irradiation as well as the rheology features. The therapeutic effects of the Cu_2_MnS_2_ nanoplates and the hydrogel were evaluated qualitatively and quantitatively in 4T1 mouse breast cancer cells. The retention, photothermal efficacy, therapeutic effects and systemic toxicity of the hydrogel were assessed in tumor bearing mouse model.

**Results:**

The Cu_2_MnS_2_ nanoplates with a diameter of about 35 nm exhibited satisfying serum stability, photo-heat conversion ability and repeated laser exposure stability. The hydrogel encapsulation did not negatively influence the above features of the photothermal agent. The nanoplates loaded in situ hydrogel shows a phase transition at body temperature and, as a result, a long retention in vivo.

**Conclusions:**

The photothermal agent embedded hydrogel played a promising photothermal therapeutic effects in tumor bearing mouse model with low systemic toxicity after peritumoral administration.

## Background

In the past few years, the world has witnessed many new methods in treating cancers [1–10], such as monoclonal antibodies, gene therapy [4, 10], photodynamic therapy (PDT), sonodynamic therapy, photothermal therapy (PTT) [8]. However, cancer therapy is still a big challenge, with the mean survival length of cancer patients only several years.

As a traditional dosage form, hydrogel has been extensively investigated in many research fields, especially in regeneration medicine. For example, adipose-derived stem cells were encapsulated in a tri-layer three-dimensional hydrogel and, the scaffold promoted bladder reconstruction by enhancing angiogenesis, innervation and smooth muscle regeneration [11]. Loading insulin and L929 fibroblasts in pH and glucose dual-responsive hydrogels could enhance collagen deposition, neovascularization, and finally promote the wound healing process in diabetic rat model [12]. Zhao et al. used phenylboronic acid-based polymeric hydrogel as the carrier of insulin and, the hydrogel exhibited the glucose-sensitive release of insulin [13]. There is a special kind of self-healing hydrogels, which exhibit similar strain-stiffening behavior and nanomechanics of biological tissues [14, 15]. Some of them are skin inspired, with pressure sensitivity and stretchability. For example, a double network hydrogel constructed by ionically crosslinked κ-carrageenan with a covalently crosslinked polyacrylamide exhibited ultra-stretchable and self-healing properties, and could be used as strain sensor [16]. Application of the hydrogels in treating cancers is also a newly emerging research field. Temperature-sensitive doxorubicin micelle which was able to form in situ hydrogels was intratumoral administered [17].

Nowadays, there has been an increasingly widespread interest in PTT. The photothermal agents (PTA) are able to convert laser energy, especially the near infrared light (NIR) which could penetrate deep into tissues, into heat energy. Up to now, PTT is often used to treat cancers. Du et al. suggested tocopherol glycol succinate functionalized Cu_3_BiS_3_ nanocrystals with strong absorption in the second biological window, the nanocrystals were used for X-ray computer tomography imaging and optoacoustic tomography imaging guided PTT [18]. Wang et al. [19] proposed shape-controlled copper selenide nanoparticles prepared by one-pot solution synthesis as a promising PTA candidate. Graphene oxide/black phosphorus nanoflakes also exhibited satisfying photothermal property [20]. Hyaluronic acid decorated gold nanorods (GNR) was reported to carry diclofenac and, diclofenac enhanced PTT of the carrier by hindering glucose uptake, blocking glycolysis, reducing adenosine triphosphate levels and finally hampering heat shock protein expression [21].

Normally, the PTA are intravenous administered to play the therapeutic effects. Despite great advances in PTT, the toxicity of the intravenous administered PTA remains a big concern as most of the PTA are made of heavy metal elements, such as gold and bismuth, that are difficult to tackle with. In addition, despite the enhanced penetration and retention effects (EPR) and other targeting methods, the nano-carriers finally distributing in tumor tissues account for only a small proportion of the dose administered, as a result, the unsatisfactory distribution retards superior therapeutic effects and increases systemic toxicity.

Indocyanine green (ICG), a typical PTA belonging to the cypates, shows severe light-bleach and reduced photothermal efficacy after repeated NIR exposure [22, 23]. Despite its excellent photo-heat conversion ability, the photothermal instability hampered the practical use of ICG as PTA. Compared to the cypates, metal nanoparticles show much higher photo-stability.

Take into account the above, in this study, an injectable Pluronic F127 hydrogel embedding copper manganese sulfide (Cu_2_MnS_2_) nanoplates for peritumoural administration is proposed (Fig. 1). Pluronic F127 is widely used in constructing thermosensitive hydrogel and, is often employed in drug delivery systems for i.v. administration [24–26]. As the hydrogel is locally administered and has a long retention time, it is believed that this system will exhibit better photothermal therapeutic effects and reduced systemic toxicity. As far as we know, PTA loaded hydrogel for cancer therapy was rarely reported.

**Fig. 1:** Schematic illustration

## Methods

### Materials

CuCl_2_·2H_2_O, MnCl_2_·4H_2_O, polyvinylpyrrolidone (PVP, M.W. 24000), Na_2_S·9H_2_O, ethylene glycol, propidium iodide, Hoechst 33342, 1,1-dioctadecyl-3,3,3,3-tetramethylindotricarbocyanine iodide (DiR) and 3-(4,5-dimethyl-2-thiazolyl)-2,5-diphenyl-2-H-tetrazolium bromide (MTT) were purchased from Aladdin (Shanghai, China). Pluronic F127 was kindly gifted by Basf (Shanghai, China).

### Preparation and characterization of Cu_2_MnS_2_ nanoplates

42 mg of CuCl_2_·2H_2_O, 31 mg of MnCl_2_·4H_2_O and 100 mg of polyvinylpyrrolidone (PVP, M.W. 24000) were added into 5 ml of ethylene glycol, the mixture was stirred to get clear solution. Then, 58 mg of Na_2_S·9H_2_O was added with stirring. The solution was stirred for 2 h to get dark brown solution. The solution was heated to 120 °C for 6 h with stirring to get dark green nanodispersions. After dialysis in deionized water for 24 h (cutting molecular weight 3000), Cu_2_MnS_2_ nanoplates was obtained. Appearance of the nanoplate was pictured by transmission electron microscopy (TEM, Shimadzu JEM-2100, 300 kV) and, the selected area electron diffraction (SAED) image was also obtained. The particle size was measured by particle sizing system (Malvern Zetasizer Nano). The concentration of Cu_2_MnS_2_ nanoplates was measured by atomic absorption spectroscopy (Shimadzu AA6800).

To investigate stability of the Cu_2_MnS_2_ nanoplates, serum was added to Cu_2_MnS_2_ nanodispersions for a final concentration of 10%, and the concentration of Cu_2_MnS_2_ nanoplates according to Cu_2_MnS_2_ was 0.1 mg/ml. The sample was placed in water bath at 37 °C for 3 days, visible absorption curves of the sample before and after storage were measured (Biotek Epoch).

To evaluate the photothermal performance of Cu_2_MnS_2_ nanoplates, the nanodispersions with different concentrations (0, 50, 100, 200 µg/ml) were exposed to 808 nm laser at 1 W/cm^2^ for 5 min. Temperatures of the samples at different time points were recorded by infrared imaging camera (Fotric 600).

To further characterize the Cu_2_MnS_2_ nanoplates, the sample with 0.1 mg/ml Cu_2_MnS_2_ was exposed to NIR irradiation for five cycles. After each irradiation for 5 min at 1 W/cm^2^, the sample was cooled to room temperature naturally, and then exposed to 808 nm laser again. Temperatures of the sample were monitored. Particle size and visible absorption curves of the sample before and after 5-cycle irradiation were measured.

### Preparation and characterization of Cu_2_MnS_2_ nanoplates embedded Pluronic F127 hydrogel

Pluronic F127 granules were simply added to Cu_2_MnS_2_ nanodispersions with stirring in ice bath to get Cu_2_MnS_2_ nanoplates loaded hydrogel. The concentration of Pluronic F127 was 0.2 g/ml and, the concentration of Cu_2_MnS_2_ nanoplates was 0.25 mg/ml.

Cu_2_MnS_2_ nanoplates loaded hydrogel was frozen in liquid nitrogen overnight, then the frozen hydrogel was lyophilized. Morphous of the final sample was viewed by scanning electron microscopy (SEM, Shimadzu SSX-550, 3.0 kV). Blank Pluronic F127 hydrogel was used as a control.

To investigate the photothermal performance of Cu_2_MnS_2_ nanoplates loaded hydrogel, the hydrogel was exposed to 808 nm laser at 1 W/cm^2^ for 5 min. Temperatures of the hydrogel at different time points were monitored. Blank hydrogel was used as a control.

To further characterize the Cu_2_MnS_2_ nanoplates loaded hydrogel, the rheology features of the samples were measured. The frequency was 1 Hz and, the heating rate was 1 °C/min (ThermoFisher-haake). The blank hydrogel was used as a control.

To study the stability of Cu_2_MnS_2_ nanoplates loaded hydrogel, the sample was placed at 37 °C for 8 days. The hydrogel sample before and after storage was diluted by water for ten times, and then measured by particle sizing system to reflect the size of the Cu_2_MnS_2_ nanoplates. Moreover, the heating curves upon NIR irradiation (808 nm, 1 W/cm^2^) were gathered before and after different storage time. The similarity between two curves was evaluated by f_2_ factor according to the following equation and, f_2_ > 50 means highly similar.

$$ f_{2} = 50\log_{10} \left\{ {\left[ {1 + \frac{1}{n}\sum\limits_{i = 1}^{n} {W_{t} } \left( {\bar{R}_{t} - \bar{T}_{t} } \right)^{2} } \right]^{ - 0.5} \times 100} \right\} $$

R_t_ and T_t_ mean temperature of the sample before and after storage upon NIR irradiation at t minute.

### Assessment of in vitro photothermal therapeutic effects

4T1 mouse breast cancer cells (1 × 10^4^) were seeded in 96-plate and incubated overnight (37 °C, 5% CO_2_), dulbecco’s modified eagle medium was used. Then, Cu_2_MnS_2_ nanodispersion was added to make final concentration of the nanoplates 0, 2, 5, 10, 20, 50 µg/ml, respectively. The cells were incubated for another 24 h. Then, the cells were exposed to 808 nm laser (1 W/cm^2^) for 1 min and, the cells free from NIR treatment were used as control. After incubation for another 4 h, the viability of the cells was measured by MTT method at 490 nm (Biotek Epoch).

4T1 mouse breast cancer cells (5 × 10^4^) were seeded in 24-plate and incubated overnight (37 °C, 5% CO_2_). Then, Cu_2_MnS_2_ nanodispersion was added to make final concentration of the nanoplates 50 µg/ml. Then, the cells were exposed to 808 nm laser (1 W/cm^2^) for 3 min and, the cells treated by PBS and the cells free from NIR treatment were used as controls. After incubation for another 4 h, propidium iodide (final concentration 30 µg/ml) was added and incubated for 30 min to stain the dead cells. Then, the culture media was discarded and the cells were washed by PBS for three times. 4% paraformaldehyde solution was used to fix the cells. After washing by PBS for three times, Hoechst 33342 solution was used to stain the nucleus of all the cells. At last, the cells were photographed by fluorescence microscope to view the photothermal therapeutic effects of the nanoplates (Leica DMi8).

4T1 mouse breast cancer cells (5 × 10^4^) were seeded in 24-plate in 1 ml of culture media. 200 µl of the Cu_2_MnS_2_ nanoplates embedded hydrogel or blank hydrogel was added to the upper transwell (8 µm). The cells were incubated at 37 °C for 24 h. Then, the hydrogels encapsulated transwells were exposed to 808 nm laser (1 W/cm^2^) for 3 min and, the cells treated by blank hydrogel and the cells free from NIR treatment were used as controls. Finally, the cells were treated and pictured as the above section.

The GreenNuc regent (Beyotime, China) was used to indicate the expression of caspase 3/7 in Cu_2_MnS_2_ nanoplates treated cells. In detail, 4T1 mouse breast cancer cells (1 × 10^4^) were seeded in 96-plate and incubated overnight (37 °C, 5% CO_2_). Cu_2_MnS_2_ nanoplates were added to the cells to make the final concentration of 50 µg/ml. The cells were further incubated for 24 h. Then, the cells were exposed to 808 nm laser (1 W/cm^2^) for 1 min and, the cells free from NIR treatment were used as control. The GreenNuc regent was added to the cells (5 µM) and incubated for 0.5 h to stain the nucleus of the caspase 3/7 expressed cells. Hoechst 33342 was also employed to stain the nucleus. Fluorescence images were captured by microscopy (Leica).

### Retention of the hydrogels around tumor tissue

The study was approved by Ethics Committee of Guangzhou Medical University.

The near infrared fluorescent dye DiR labeled hydrogel was prepared by adding DiR ethanol solution (100 µg/ml) to the blank hydrogel with stirring in ice bath to make the final concentration of 5 µg/ml. The control DiR solution was prepared by adding DiR ethanol solution (100 µg/ml) to PBS with stirring to make the same final concentration of 5 µg/ml before use.

At day 0, Balb/c mouse (female, 6–8 week old) was subcutaneously administered 1 million of 4T1 cancer cells to establish armpit tumor bearing mouse model. At day 10, 200 µl of DiR labeled hydrogel was peritumoral injected. Mice received 200 µl of the DiR solution were used as control. Then at different time intervals, the DiR signals were captured at 740/820 nm to image the retention of the hydrogels around tumor tissue (Berthold NightOWL LB983).

### In vivo anti-cancer performance

The study was approved by Ethics Committee of Guangzhou Medical University.

At day 0, Balb/c mouse (female, 6–8 week old) was subcutaneously administered 1 million of 4T1 cancer cells to establish armpit tumor bearing mouse model. At day 7, the volume of the tumor reached approximately 200 mm^3^ according to the following equation: volume = length × (width)^2^/2. Then, 200 µl of the Cu_2_MnS_2_ nanoplates loaded hydrogel was administered by peritumoral injection. Mice received 200 µl of the blank hydrogel were used as control. After 2 h, the tumors were exposed to 808 nm laser at 1 W/cm^2^ for 5 min after the mice were anesthetized. Temperatures of the tumor tissues were recorded by infrared imaging camera. NIR treatment was carried out every day from then on. At day 15, the mice were sacrificed and, the tumors of the test and control group were photographed and weighed. Then, the tumor samples were made into paraffin sections and H&E stained. The main organs of heart, liver, spleen, lung and kidney were also sliced and H&E stained. Body weight of the mice was measured everyday.

### Elimination

Cu_2_MnS_2_ nanoplates (200 µg/ml, 200 µl) in saline were i.v. injected into healthy mice. Three hours later, the urine was collected and measured by the particle sizing system. The urine collected before treatment was used as a control.

### Statistical analysis

All values were expressed as mean ± standard deviation (SD). All comparisons were performed by the two-tailed Student’s *t* test. A *p*-value less than 0.05 was supposed to be statistically significant and, *p*-value less than 0.01 was considered to be highly significant.

## Results and discussions

### Characteristics of the Cu_2_MnS_2_ nanoplates

The Cu_2_MnS_2_ nanoplatform was prepared by a simple one-pot synthesis. PVP was used as the stabilizer of the nanodispersions due to its favourable hydrophilicity. The final product appeared to be a dark green solution and, the concentration of the nanoplatform could be simply adjusted by dilution through adding deionized water.

Figure 2a (upper) shows that Cu_2_MnS_2_ existed as irregular nanoplates in the solution, with a diameter of approximately 30 nm. Particle size of the nanoplates was further validated by particle sizing system (Fig. 2b), which shows a single peak around 35 nm. The appearance and size of the Cu_2_MnS_2_ nanoplates were in accordance with other reports [27]. The SAED image in Fig. 2a (lower) indicates that the Cu_2_MnS_2_ nanoplates were in the form of polycrystals.

**Fig. 2:** In vitro characterization of the Cu_2_MnS_2_ nanoplates. **a** TEM and SAED images of the Cu_2_MnS_2_ nanoplates; **b** the particle size of the Cu_2_MnS_2_ nanoplates; **c** the visible absorption curves of Cu_2_MnS_2_ nanoplates before and after incubation in serum for 3 days at 37 °C; **d** and **e** the thermographs and corresponding heating curves of the Cu_2_MnS_2_ nanoplates at varied concentrations upon 808 nm laser exposure (1 W/cm^2^); **f** the heating curves of the Cu_2_MnS_2_ nanoplates upon repeated 808 nm irradiation (1 W/cm^2^); **g** particle sizes of the Cu_2_MnS_2_ nanoplates before (green) and after (red) 5-cycle 808 nm irradiation (1 W/cm^2^); **h** the visible absorption profiles of the Cu_2_MnS_2_ nanoplates before and after 5-cycle 808 nm irradiation (1 W/cm^2^)

The NIR is considered to be biologically compatible due to its deep tissue penetration and negligible influence on tissues. PTAs are able to convert the light to heat to exhibit anti-cancer effects by generating intolerable high temperature microenvironment for malignant cells. The light-heat conversion ability of the PTAs can be indicated by visible absorption curve. The visible absorption curve in Fig. 2c saw a steady increase from 550 to 1000 nm, implying the encouraging NIR absorption capacity.

The stability of PTA in the body fluids is critical for its performance in vivo. To assess the stability of the PTA, the visible absorption curve of the Cu_2_MnS_2_ nanoplates exposed to 10% blood serum for 3 days at 37 °C was compared to that of the original sample. The sample after serum exposure still exhibited an increasing visible absorption curve, which was highly comparable to the original one (Fig. 2c). The similar two curves clued the outstanding stability of the Cu_2_MnS_2_ nanoplates in body fluids and, as a result, promising photothermal performance in vivo.

Figure 2d and e show the thermo-photographs and heating curves of the Cu_2_MnS_2_ nanoplates with a serial concentrations of 50, 100, 200 µg/ml upon 808 nm laser exposure. The Cu_2_MnS_2_ nanoplates exhibited dramatic increase in temperature upon NIR irradiation at any concentration. Moreover, the temperature rises along with the increase of concentration, with the final temperature of the three concentrations reaching 52.1, 59.8, 62.6 °C, respectively. Meanwhile, the NIR exposure did not make any changes to the temperature of deionized water. In a word, the above results indicated the favorable photothermal effects of the Cu_2_MnS_2_ nanoplates.

Photothermal stability is one of the most important index to assess PTA. As the Cu_2_MnS_2_ nanoplates loaded hydrogel would be locally administered, it was hoped that the PTA in the formed hydrogel would be able to exert long-term therapeutic effects. Figure 2f shows the heating curve of the Cu_2_MnS_2_ nanoplates upon repeated NIR irradiation. The nanodispersion could be re-heated to about 60 °C after 5 min laser exposure once the sample was naturally cooled to room temperature. In other words, the heating curve of each cycle was identical to the other ones, with the highest temperature of each cycle nearly 60 °C, and the heating curve showed negligible changes after repeated laser exposure. These data indicated that the Cu_2_MnS_2_ nanoplates displayed satisfying photothermal stability. To further validate this feature, the particle size and visible absorption curve of the nanoplates before and after 5-cycle NIR irradiation were measured. Figure 2g shows that the particle size of the sample post-NIR treatment was about 31 nm, slightly smaller than the diameter of 35 nm before NIR treatment. Figure 2h shows that the two visible absorption curves of the nanoplates were obviously identical, with minor variations. Both graphs further support the encouraging photothermal stability of the Cu_2_MnS_2_ nanoplates. Based on these results, it is estimated that the PTA would maintain the therapeutic effects throughout the whole retention period in vivo and would not be destroyed by body fluids or repeated laser exposure.

### Features of the Cu_2_MnS_2_ nanoplates loaded Pluronic F127 hydrogel

For the purpose of reducing the systemic toxicity of the intravenously administered PTA and overcoming the possible problem of unsatisfying photothermal therapeutic effects due to the limited enrichment of the PTA in tumor tissues, thermosensitive in situ hydrogel was employed to encapsulate the Cu_2_MnS_2_ nanoplates, which would be peritumorally injected. It was believed that the injectable hydrogel would solidify locally and, form semisolid hydrogel surrounding the tumor tissue and, might exhibit a long retention time. Meanwhile, the local administration would decrease systemic toxicity and increase therapeutic outcomes. In this section, the in vitro characteristics associated with the above aims would be discussed in detail.

The Cu_2_MnS_2_ nanoplates embedded hydrogel was prepared by a simple one-pot method of dissolving Pluronic F127 in the nanodispersions directly. Figure 3a shows the morphous of the blank hydrogel and the PTA encapsulated hydrogel. Both hydrogels had a highly macroporous network structure, with the pores about 50–200 µm in diameter. In detail, the blank hydrogel shows more but smaller pores than the Cu_2_MnS_2_ nanoplates embedded hydrogel. With 10,000-fold magnification, the blank hydrogel displayed a smooth surface, while the surface of the Cu_2_MnS_2_ nanoplates embedded hydrogel was noticeably rough. Actually, there were many nanoparticles evenly dispersed in the hydrogel matrix. The nanoparticles were about tens of nanometers in diameter, corresponding well to the size of the Cu_2_MnS_2_ nanoplates. It was supposed that the PTA dispersed evenly in the hydrogel matrix.

**Fig. 3:** In vitro characterization of the Cu_2_MnS_2_ hydrogel. **a** SEM images of the blank Pluronic F127 hydrogel and the Cu_2_MnS_2_ nanoplates loaded hydrogel; **b** and **c** the thermographs and corresponding heating curves of the Cu_2_MnS_2_ hydrogel and blank hydrogel upon 808 nm irradiation (1 W/cm^2^); **d** pictures of the blank hydrogel and Cu_2_MnS_2_ hydrogel at 4 and 37 °C; **e** the complex viscosity and loss modulus curves of the blank hydrogel and Cu_2_MnS_2_ hydrogel; **f** particle size of the Cu_2_MnS_2_ nanoplates encapsulated in the hydrogel after different storage time at 37 °C; **g** the heating profiles of the Cu_2_MnS_2_ hydrogel upon 808 nm laser exposure (1 W/cm^2^) after different storage time at 37 °C

Ideally, the Cu_2_MnS_2_ nanoplates embedded hydrogel would exhibit pronouncing photothermal performance. Figure 3b and c show the temperature changes of the PTA encapsulated hydrogel and the blank control hydrogel upon 808 nm laser exposure. The temperature of the Cu_2_MnS_2_ hydrogel increased dramatically to 62.2 °C upon NIR irradiation. The heating curve of the Cu_2_MnS_2_ hydrogel shown in Fig. 3c was comparable to that of the nanodispersions illustrated in Fig. 2e. Moreover, the laser exposure had little influence on the blank hydrogel, with negligible temperature changes throughout the whole period. It was concluded that the encapsulation in hydrogel did not negatively influence the photothermal performance of the Cu_2_MnS_2_ nanoplates and, the nanoplates loaded hydrogel was supposed to display excellent photo-heat conversion transition capacity in vivo.

To elevate the compliance of the patients, non-invasive treatment is highly required nowadays. Injectable hydrogel is one of the most widely used non-invasive administration route. Pluronic F127 is a commercially available thermosensitive hydrogel constructing material. Figure 3d shows that both the blank hydrogel and the Cu_2_MnS_2_ hydrogel are liquid at 4 °C and, the two hydrogels changed into semisolid at body temperature. In other words, the formed in situ hydrogel maintained its fluidity at low temperature (< 20 °C) and, the fluidity assigned the injectable feature of the hydrogel. At the same time, the in situ hydrogel solidify at body temperature and, the semisolid state would promise a long retention time in vivo. To explain the phase transition of the hydrogels in detail, the rheology characteristics of the hydrogels were studied. Figure 3e (upper) shows the complex viscosity of the blank hydrogel and the Cu_2_MnS_2_ hydrogel. Both of the curves exhibited a sharp increase in the complex viscosity in a narrow temperature range. In detail, the complex viscosity profile of the blank hydrogel saw a phase transition temperature of 30 °C, while the encapsulation of the Cu_2_MnS_2_ nanoplates resulted in a decrease in phase transition temperature to 27 °C. The loss modulus curves in Fig. 3e (lower) displayed the same transition temperatures. Normally, loading water-soluble substances will increase the phase transition temperature of the hydrogel, while embedding water-insoluble agents will decrease the phase transition temperature. Despite the water-soluble PVP in the nanoplates, the Cu_2_MnS_2_ core was water-insoluble and hydrophobic. As a result, there was a reduction in the phase transition temperature of the hydrogel after the Cu_2_MnS_2_ nanoplates encapsulation. Anyhow, it can be concluded that the Cu_2_MnS_2_ hydrogel would undergo a phase transition process after being locally administered, assigning the hydrogel a long retention time in vivo.

One of the advantage of the injectable hydrogel in treating cancers is the sustained therapeutic efficacy. To achieve this, the PTA in the hydrogels must be stable for a considerable period. In this research, the particle size and the heating curve of the Cu_2_MnS_2_ nanoplates after being encapsulated were measured. Figure 3f shows that the nanoplates in the hydrogel maintained a nearly constant diameter around 40 nm, comparable to the original particle size before being loaded. The slight size increase was probably due to the adsorption of Pluronic F127 on the surface of the Cu_2_MnS_2_ nanoplates. The result indicated that the Cu_2_MnS_2_ nanoplates remained stable in the hydrogel in the term of particle size. Figure 3g shows the heating profiles of the Cu_2_MnS_2_ hydrogel before and after storage at 37 °C for several days. It can be seen that all the heating curves were similar, with the temperature reaching about 60 °C at the end of laser exposure. It seems that the encapsulation and storage at body temperature had little influence on the photothermal performance of the Cu_2_MnS_2_ nanoplates. What’s more, as all the heating profiles were obtained by recording the thermograph of the same hydrogel sample upon NIR irradiation at different time intervals, it can be concluded that the Cu_2_MnS_2_ nanoplates remained stable in photo-heat transition ability after repeated 808 nm laser exposure. Statistically, the similarity factor f_2_ between the initial heating curve and that of the 4th, 6th, 8th day were 76.2, 70.5 and 70.7, respectively. All the similarity factor f_2_ is over 50, which represented that all the heating profiles were highly comparable. In a word, both results supported that encapsulation in the hydrogels and storage at body temperature would not negatively influence the Cu_2_MnS_2_ nanoplates and, implied that the PTA would perform sustained therapeutic effects in vivo.

### In vitro anti-cancer photothermal therapy

In this section, the photothermal therapeutic effects of the Cu_2_MnS_2_ nanoplates and the PTA loaded hydrogel against the 4T1 mouse breast cancer cells were evaluated.

Figure 4a illustrates the fluorescence images of the 4T1 cells, with all the cells blue stained and the dead cells red stained. As anticipated, the PBS treatment alone resulted in few cell death, with negligible number of the cells red stained. What’s more, the combination of PBS treatment and 808 nm laser exposure also led to insignificant cell death, with only a few cells red stained. The results indicated that the NIR light did not make detrimental effects on the cell survival and, the NIR light could be regarded as bio-safe to some extents. Furthermore, the Cu_2_MnS_2_ nanoplates at the concentration of 50 µg/ml did not exert obvious toxicity to cells, as implied by the comparable extent of cell death compared to the PBS control group. The result clued the encouraging biocompatibility of the Cu_2_MnS_2_ nanoplates. Based on the observation, it was believed that the PTA would produce tolerable side effects to healthy tissues without NIR irradiation. As anticipated, the combination of Cu_2_MnS_2_ nanoplates treatment and 808 nm laser exposure resulted in significant cell deaths, with almost all the cells under irradiation failed to survive. Moreover, the overlay image shows a clear dividing line separating the alive and dead cells. Actually, the dividing line was the boundary of the laser light, merely the cells covered by the laser light were sentenced to death. The existence of the dividing line pointed out that the photothermal therapy could be carried out accurately and precisely.

**Fig. 4:** The anti-cancer effects of the Cu_2_MnS_2_ nanoplates and the hydrogel against 4T1 mouse breast cancer cells. **a** The fluorescence images of the 4T1 cells after being treated by the Cu_2_MnS_2_ nanoplates differently, the red color represents the dead cells stained by propidium iodide and the blue color represents the nucleus of all the cells, the white line is the boundary of the 808 nm laser; **b** the survival rates of the 4T1 cells measured by MTT test after being treated by the Cu_2_MnS_2_ nanoplates differently, ** represents statistically high significance (*p* < 0.01); **c** the fluorescence images of the lower 4T1 cells after being treated by the blank hydrogel and Cu_2_MnS_2_ hydrogel in the upper transwell differently, the red color represents the dead cells stained by propidium iodide and the blue color represents the nucleus of all the cells; **d** the caspase 3/7 expression of the Cu_2_MnS_2_ nanoplates treated cells, the green-stained nucleus indicate the cell apoptosis

To analyze the toxicity and therapeutic effects of the Cu_2_MnS_2_ nanoplates quantitatively, MTT test was carried out. Figure 4b shows the 4T1 cancer cell survival rate after being differently treated. When the cells were free from the laser exposure and treated by the Cu_2_MnS_2_ nanoplates for 24 h only, the viability of the cells saw a decreasing trend along with the PTA concentration increase, with the survival rate declining to 85.7%, 75.1% and 60.2% at the Cu_2_MnS_2_ nanoplates concentration of 10, 20, 50 µg/ml, respectively. Once the cells treated by the Cu_2_MnS_2_ nanoplates at the same concentrations were exposed to laser light, the viability of the cells further declined to 52.5%, 33.1% and 12.6%. The NIR exposure made statistically significant difference to the survival rate of the Cu_2_MnS_2_ nanoplates treated cells when the PTA concentration reached 10, 20 and 50 µg/ml. Above results clued that the Cu_2_MnS_2_ nanoplates treatment plus the NIR irradiation would exert dramatic harm to the cancer cells and, the malignant cells could be totally wiped out at a high PTA concentration. As a result, it can be anticipated that the enrichment of the Cu_2_MnS_2_ nanoplates surrounding the tumor tissues by local administration of the PTA encapsulated hydrogel would bring in promising therapeutic effects.

In this study, transwell was employed to examine the therapeutic effects of the Cu_2_MnS_2_ hydrogel against the 4T1 cancer cells. The transwell membrane separated the upper PTA embedded hydrogel and the lower cells. Figure 4c shows the fluorescence images of the cells, with all the cells blue stained and the dead cells red stained. It can be seen that the blank hydrogel alone did not induce cell death, indicating the outstanding compatibility of the Pluronic F127 hydrogel matrix. Moreover, the blank hydrogel plus the laser exposure did not produce cell death either. As discussed above, the NIR irradiation did not make any changes to the hydrogel. The absence of cell death when the blank hydrogel and the laser exposure were combined administered further proved this point. Figure 4c also shows that the Cu_2_MnS_2_ hydrogel alone was not harmful to the cells, with negligible number of cells red stained. It seems that, despite the same incubation time, the cells treated by the PTA loaded hydrogel exhibited much higher survival rate than the cells treated by the same amount of the nanoplates directly, as indicated in Fig. 4b. The difference implied that the encapsulation in the hydrogel reduced the unwanted adverse effects of the Cu_2_MnS_2_ nanoplates. It was supposed that the hydrogel matrix relieved the undesirable toxicity of the chemicals by “prisoning” them and, played the therapeutic effects through photo-heat conversion only. The capacity of relieving the direct toxicity caused by the metal chemicals renders the hydrogel an ideal candidate to decrease the systemic toxicity of the PTA. Figure 4c also shows that the cancer cells were almost completely wiped out when the cells were exposed to the Cu_2_MnS_2_ hydrogel together with the NIR irradiation. Obviously, the temperature rise caused by the Cu_2_MnS_2_ hydrogel under the laser exposure killed the malignant cells. It is worth noting that, despite the same irradiation time and strength as well as the PTA dose, the Cu_2_MnS_2_ hydrogel produced much bigger cell death area than the free nanoplates, as indicated in Fig. 4a. In other words, concentrated PTA played more promising photothermal therapy than the evenly dispersed PTA of the same dose. That is to say, the hydrogel not only reduced the direct chemical toxicity of the Cu_2_MnS_2_ nanoplates, but also enhanced the photothermal therapeutic effects. The phenomenon further indicated the superiority of the hydrogel in achieving more pronouncing photothermal therapy.

To further indicate the influence of Cu_2_MnS_2_ nanoplates on the malignant cells, the apoptosis was detected by the GreenNuc regent. The regent was a DNA-binding fluorescence substance linked to peptide sequence DEVD. The DEVD peptide was highly negative charged and, as a results, retards the binding of the fluorescence substance and the nucleus. Moreover, the active caspase 3/7 could identify the DEVD sequence and release the fluorescence agent. The free fluorescence substance would bind DNA and, make the nucleus green-stained. In a word, the green-stained nucleus imply the expression of caspase 3/7, a well-known apoptosis marker. Figure 4d shows that the Cu_2_MnS_2_ nanoplates treated cells displayed green-stained nucleus after the laser exposure, indicating the cell apoptosis. On the other hand, green fluorescence was not observed in the nanoplates treated only cells. In other words, the nanoplate was bio-safe and, did not harm the cells. Furthermore, the generated heat of the nanoplates upon laser exposure could induce cell apoptosis.

### Local retention of the Cu_2_MnS_2_ nanoplates loaded hydrogel

In order to reduce the systemic toxicity and enhance the photothermal therapeutic effects, the Cu_2_MnS_2_ hydrogel was peritumorally administered. It was supposed that the thermosensitive hydrogel would change into semisolid hydrogel locally, and then the encapsulated Cu_2_MnS_2_ nanoplates would have a long retention surrounding the tumor tissues and, as a result, play sustained therapeutic effects after only one non-invasive administration. The prerequisite of the sustained therapeutic effects is the long retention in vivo. To image the retention of the hydrogel in vivo, near-infrared imaging technique was employed. The near-infrared fluorescence dye DiR labeled hydrogel was used, with the DiR solution used as a control group. Figure 5a shows the fluorescence images of the breast tumor bearing mice after being peritumorally treated by DiR hydrogel or free DiR solution. The free DiR treated mice showed a rapid signal decrease, with weak fluorescence signal at day 10 and almost undetectable fluorescence signal at day 15. The fast fluorescence signal decrease meant the rapid loss of the agent from the tumor site. At the same time, the DiR hydrogel treated mice saw a nearly constant fluorescence signal, with the signal strength at day 10 comparable to the original signal strength at day 0 and only a slight signal decrease at day 15. The stable fluorescence strength indicated little loss of the agent from the tumor site. In other words, the in situ hydrogel guaranteed a promising retention of the treating agents surrounding the tumor site and, as a result, provided the basis of sustained therapeutic effects.

**Fig. 5:** In vivo performances of the Cu_2_MnS_2_ hydrogel in tumor bearing mouse model. **a** The retention of the DiR labeled hydrogel and free DiR solution after peritumoral administration (Ex/Em: 740/820 nm); **b** and **c** the thermographs and the corresponding heating curves of the tumor sites after peritumoral administration of the blank hydrogel or Cu_2_MnS_2_ hydrogel plus 808 nm irradiation (1 W/cm^2^); **d** pictures of the tumor tissues after photothermal therapy (1 W/cm^2^, 5 min) in eight sequential days, the red circle represents visibly undetectable tumor sample; **e** statistic graph of the tumor weights, * represents statistical significance (*p* < 0.05); **f** hematoxylin & eosin staining of the tumor tissues

### In vivo anti-cancer performance

In this section, the anti-cancer performance of the Cu_2_MnS_2_ nanoplates embedded hydrogel was evaluated in a breast cancer bearing mouse model, with the blank hydrogel as a control.

Figure 5b shows the thermographs of the Cu_2_MnS_2_ hydrogel or blank hydrogel peritumorally treated tumor bearing mice upon the 808 nm laser irradiation. Figure 5c illustrated the temperatures of the tumor tissue at varied time points. It can be seen that the blank hydrogel treated mouse exhibited a moderate temperature increase at the tumor site upon the NIR exposure, with the temperature reaching 45.9 °C at the end of irradiation. The temperature increase was probably caused by the direct tissue heating effect of the NIR. Meantime, the Cu_2_MnS_2_ hydrogel treated mouse displayed a sharp temperature increase at the tumor site upon the laser exposure, with the temperature approaching 90 °C at the end of NIR irradiation. The results implied the outstanding photo-heat transition ability of the PTA loaded hydrogel in vivo. The satisfying photo-heat transition capacity was supposed to promise a pronouncing photothermal therapeutic effect against cancer.

After the NIR irradiation in eight sequential days, the tumor tissues of the test and control groups were collected, as shown in Fig. 5d. Despite the same laser strength and lasting time, the tumor samples of the blank hydrogel treated mice were obviously bigger than that of the Cu_2_MnS_2_ hydrogel treated mice. Specially, two mice peritumorally treated by the Cu_2_MnS_2_ hydrogel plus the NIR irradiation were totally cured, with the tumor tissues visibly undetectable at the end of the experiment. The tumor weights between the test and control group were statistically different (*p* < 0.05), with the mean tumor weight 0.15 g and 0.76 g respectively, as illustrated in Fig. 5e. The above results indicated the excellent photothermal therapeutic effects of the Cu_2_MnS_2_ nanoplates encapsulated hydrogel against cancer.

As shown in Fig. 5f, it is worth noting that, comparable to the control group, the necrosis was absent in the tumor tissue of the test group. It was estimated that the heat generated could not penetrate into the core of the tumor tissue to induce cell death, as a result, the necrosis was undetectable in the remaining tumor tissue. The phenomenon clued that the Cu_2_MnS_2_ hydrogel played the therapeutic effects through “burning” the cancer cells layer by layer.

### Systemic toxicity and elimination of the nanoplates

To evaluate the systemic toxicity of the treatments, the body weights of the mice were measured. Figure 6a shows that the mice of both groups had a nearly constant body weight, with a small initial fluctuation probably due to the inadaptation to anesthesia in the first few days. The relatively stable body weight indicated that the non-invasive administration of the thermosensitive Cu_2_MnS_2_ hydrogel plus the laser irradiation induced negligible systemic toxicity. The main organs of heart, liver, spleen, lung and kidney (Fig. 6b) show normal morphous and, further indicated the negligible systemic toxicity of the treatment.

**Fig. 6:** Systemic toxicity evaluation and elimination of the nanoplates. **a** Body weight curves of the tumor bearing mice throughout the whole experiment period; **b** H&E staining of the main organs of the Cu_2_MnS_2_ hydrogel and the blank hydrogel treated tumor bearing mice; **c** particle sizing measurement of the urine samples of the Cu_2_MnS_2_ nanodispersions i.v. treated mice

The urine of the mice before and after i.v. administration of the Cu_2_MnS_2_ nanoplates was assessed by the particle sizing system. The urine of the treated mice displayed a single peak about 20 nm, similar to the size of the original nanoplates (Fig. 6c). At the same time, the small particle was not observed in the urine of the mice before administration. It was assumed that the peak observed in the urine corresponded to the excreted nanoplates. In other words, the Cu_2_MnS_2_ nanoplates could be eliminated by kidney excretion.

In summary, it is clear that the injectable and temperature-responsive in situ Cu_2_MnS_2_ hydrogel is a promising PTA for cancer treatment with low systemic toxicity.

## Conclusions

In this study, an injectable and thermosensitive hydrogel encapsulating Cu_2_MnS_2_ nanoparticles for photothermal therapy against cancer was reported. The Cu_2_MnS_2_ particles show nanoplate structure with a diameter of about 35 nm. The nanoplates evenly distributed in the hydrogel matrix and, maintained its particle size unchanged. The PTA loaded hydrogel shows excellent photo-heat conversion ability and outstanding repeated irradiation stability. The hydrogel not only exhibited thermo-responsive in situ gel-forming capacity at body temperature, but also reduced the chemical toxicity of the Cu_2_MnS_2_ by “prisoning” the nanoplates in the matrix. Moreover, the concentrated PTA in the hydrogel performed more promising therapeutic effects against cancer cells than the nanoplates solution. At last, the Cu_2_MnS_2_ nanoplates embedded hydrogel displayed pronouncing tumor curing effects after peritumoral administration due to the enhanced retention in vivo and elevated local temperature surrounding the tumor tissue upon the NIR exposure. Meantime, the preparation shows insignificant systemic toxicity.

## Abbreviations

Cu_2_MnS_2_: copper manganese sulfide
PDT: photodynamic therapy
PTT: photothermal therapy
NIR: near infrared light
PTA: photothermal agents
GNR: gold nanorods
EPR: enhanced penetration and retention effects
PVP: polyvinylpyrrolidone
TEM: transmission electron microscopy
SEM: scanning electron microscopy
SAED: selected area electron diffraction
